# Tissue Composition and Biomechanical Property Changes in the Vaginal Wall of Ovariectomized Young Rats

**DOI:** 10.1155/2019/8921284

**Published:** 2019-07-31

**Authors:** Meng Mao, Yaqian Li, Ye Zhang, Jia Kang, Lan Zhu

**Affiliations:** ^1^Departments of Obstetrics and Gynecology, Peking Union Medical College Hospital, Peking Union Medical College, Chinese Academy of Medical Sciences, Beijing, China; ^2^Department of Central Laboratory, Peking Union Medical College Hospital, Peking Union Medical College, Chinese Academy of Medical Sciences, Beijing, China

## Abstract

Ideal animal models are needed to reflect the changes in the biochemical and biomechanical properties of the vagina that occur in pelvic organ prolapse (POP). In this study, we aimed to demonstrate the short and long-term effect of menopause on the biochemical and biomechanical properties of rat anterior vaginas. Here, Sprague-Dawley rats were bilaterally ovariectomized to induce menopause. Rats without ovariectomy served as the normal control group (n=12). The histology changes and the expression of collagen I, III, and a-SMA were assessed to indicate the biochemical changes in the vagina 2 weeks, 4 weeks, and 16 weeks after ovariectomy (n=6 for 2 and 4 weeks, n=12 for 16 weeks). Uniaxial biomechanical testing was conducted in the control group and ovariectomized rats 16 weeks after ovariectomy. Compared with the control group, the ovariectomy group showed a significant increase in the expression of collagen I 2 weeks after ovariectomy, while collagen III showed a declining trend. Two weeks after ovariectomy, the smooth muscle bundles began to become disorganized, and the fraction of smooth muscle in the nonvascular muscularis of the proximal vagina was significantly decreased (P<0.001). However, there was no difference in the expression of a-SMA in the distal vagina. Compared with the control group, the ovariectomy group had stiffer vaginas with a declining trend in the ultimate load 16 weeks after ovariectomy. In conclusion, surgically induced menopause had a significant short- and long-term impact on tissue composition and biomechanical properties of the rat vagina, which may lead to increased susceptibility to POP development.

## 1. Introduction

Pelvic organ prolapse (POP) refers to the herniation of pelvic organs, including the uterus, bladder, small bowel, and rectum, into the vaginal cavity. POP affects almost 50% of postmenopausal women [1]. Despite its high prevalence and significant impact on the quality of life, the pathophysiology of prolapse remains poorly understood. The normal positions of pelvic organs are supported by a normally supported vagina [2]. Therefore, a structural defect in the vagina and its supportive tissues is thought to be involved in the development of POP [3, 4].

The vaginal wall comprises the following four layers: epithelium, lamina propria, muscularis, and adventitia [5]. The lamina propria is a dense connective tissue layer composed primarily of collagen and elastin. The muscle layer mainly contains smooth muscle. Together, the two layers confer the greatest tensile strength to the vaginal wall. Collagen I and collagen III are the predominant extracellular matrix components and significantly contribute to the biomechanical properties of the vagina [6]. Collagen I and collagen III have different fiber diameters, resulting in differences in their mechanical properties. Collagen I provides tensile strength and stiffness, while collagen III prevails in more flexible tissue [7, 8]. Previous studies have focused on the differences in vaginal biopsies between patients with and without POP, and a disequilibrium between collagen I and collagen III and a decreased fraction of smooth muscle have been found in prolapsed vaginal tissues [9–11]. These changes can compromise the biomechanical properties of the vagina, even leading to the development of POP. Tissue engineering may provide novel approaches for the treatment of POP by restoring the collagen subtype ratio and smooth muscle content in the vagina.

To develop new treatments for POP, an appropriate animal model that reflects the changes in the vagina that occur in human POP is needed. The structural properties of the vagina and its supportive tissues in rats have been shown to be similar to those in humans [12]. Several studies have focused on the impact of pregnancy and vaginal delivery on the biomechanics of the rat vagina and had similar findings [13, 14]. Compared to virgin rats, the linear stiffness of the vagina appeared to decrease during the stages of pregnancy and immediately after delivery. However, the injuries caused by vaginal delivery are recoverable because the vaginal linear stiffness returned to a normal level after 4 weeks postpartum. Therefore, the rat model of vaginal delivery alone is not ideal. In addition to vaginal delivery, aging is another major risk factor for POP [15]. The prevalence of prolapse increases with advancing age, and most women do not develop prolapse until years after their first delivery [16]. However, few studies have examined the alteration in the structure components and biomechanical properties of the rat vagina after menopause [17, 18].

In this study, we used ovariectomized rats as a model of surgical menopause. The main objective of this study was to delineate the short- and long-term effects of menopause on the collagen content, collagen subtypes, smooth muscle content, and biomechanical property changes in the vagina.

## 2. Materials and Methods

### 2.1. Animals

The use of Sprague-Dawley (SD) rats and the experimental procedures were approved by the Institutional Review Board of Peking Union Medical College Hospital (PUMCH), Beijing, China. The “Guidance suggestions for the care and use of laboratory animals” (Ministry of Science and Technology of the People's Republic of China, 2006) were followed. Thirty-six female SD rats aged 8 weeks (205±15 g) were provided by the laboratory animal unit of PUMCH. To control for the effects of parity, all rats were virgins. The rats were raised under standard laboratory conditions (temperature 20-22°C, relative humidity 50-70%, 12 h/12 h light/dark cycle) and received food and water ad libitum. The animals were housed for 2 weeks before starting the experiment to allow time to acclimate.

### 2.2. Experimental Design

In total, 36 SD rats were randomly assigned to the following 4 groups: in Group 1 (control group), the animals were sacrificed and tested without any intervention at baseline (12 subjects, including 6 for the biomechanical testing); in Group 2, the animals were sacrificed 2 weeks after bilateral ovariectomy (6 subjects); in Group 3, the animals were sacrificed 4 weeks after bilateral ovariectomy (6 subjects); and in Group 4, the animals were sacrificed 16 weeks after bilateral ovariectomy (12 subjects, including 6 for the biomechanical testing).

On the first day of the study, the animals in all groups (except for Group 1) were bilaterally ovariectomized to clearly define the menopausal status. All operations were performed by one surgeon. The animals were anesthetized by an intraperitoneal injection of 1% pentobarbital sodium (0.4 mL/100 g). Ovariectomy was performed through a 2 cm ventral midline incision in the upper abdomen under sterile conditions. The ovaries were well exposed and excised. Then, the muscle wall and skin were closed with interrupted sutures by Mersilk 4-0 (Ethicon, USA). Penicillin was administered to each animal to prevent infection after the operation. On the first day of the study and 2, 4, and 16 weeks after ovariectomy, 12 (Group 1), 6 (Group 2), 6 (Group 3), and 12 (Group 4) rats, respectively, were sacrificed under complete anesthesia for the anterior vaginal wall tissue collection. Our decision to sacrifice the rats at 2 weeks was based on a previous study that demonstrated that surgically induced anestrus starts 15 days after surgery based on the pre- and postsurgery estradiol levels [19].

### 2.3. Tissue Preparation

After euthanasia, we opened the abdominal cavity and disarticulated the pubic symphysis. First, the vaginal orifice was isolated from the surrounding perineal skin. Then, the vaginal tube was isolated intact and dissected from the connective tissue, bladder, urethra, and cervix. The perineal skin was removed. The freshly harvested vaginal tube tissue was cut longitudinally, and the anterior vaginal wall was collected for testing. We cut the anterior vaginal wall transversely into proximal (approximately upper two-thirds) and distal (approximately lower one-third) segments. The proximal segment was immediately immersed in 10% neutral buffered formalin, processed, and embedded in paraffin blocks for the histology and immunohistochemistry analyses. The distal segment was snap-frozen in liquid nitrogen and stored at -80°C for the molecular studies. In total, 6 rats were included in the biomechanical testing of Group 1 and Group 4. The anterior vaginal wall was collected as described above, wrapped in wet gauze moistened with 0.9% normal saline, and stored at 0-4°C in a refrigerated box. Biomechanical testing was performed within 4 h of harvesting the tissue.

### 2.4. Histology/Immunohistochemistry

#### 2.4.1. Masson Trichrome Staining

For each animal, a 5-*μ*m-thick cross-section of a paraffin-embedded proximal vaginal segment (n=6 animals/group) was stained with Masson trichrome stain (MTS) for the morphological examination. The images of the MTS sections were visualized under a Nikon Eclipse CI microscope and captured with a Nikon DS-U3 camera.

#### 2.4.2. Picro-Sirius Red Staining

Sirius Red birefringence was used to assess the percent area of both immature and mature collagen fibrils in the lamina propria of the proximal vaginal segment. After dewaxing and rehydrating in graded alcohols, 5-*μ*m-thick cross-sections were stained with Picro-Sirius Red using previously established protocols [20]. Briefly, the slides were stained with Sirius Red F3B (0.1 g/100 mL saturated picric acid solution) (Sigma-Aldrich, USA) for 1 h at room temperature. Then, the stained slides were washed with running water (nonacidified) to remove the yellow picric acid counterstain. Six images at 20X magnification per slide were taken of the lamina propria regions under a Nikon Eclipse CI light microscope equipped with a polarizing filter to identify the birefringent Sirius Red-stained collagen fibers. The images were examined using Image-Pro Plus Version 6.0 software by identifying thicker mature (orange/red colored) and thinner immature (green colored) collagen fibers. Three slides were cut transversely from different portions along the vagina longitudinal axis per animal. The thicker and thinner fibers were measured as the percentage area of the lamina propria in six images per slide. These replicates were averaged per animal and used to obtain the means of each group (n=6 animals/group).

#### 2.4.3. a-SMA Immunohistochemistry

Five-micron-thick cross-sections of the paraffin-embedded proximal vaginal segment were immunohistochemically processed for the detection of a-SMA. The slides were deparaffinized in xylene, rehydrated through a graded series of ethanol, and washed with distilled water. The antigens were retrieved by incubating the slides in citrate buffer (pH 6.0) in a water bath at 95-100°C for 20 min. The slides were cooled for 15 min at room temperature and washed with PBS (3 washes of 5 min each). Then, the endogenous peroxidases were blocked with 3% H_2_O_2_ for 20 min at room temperature, and the slides were washed with PBS (3 washes of 5 min each). Then, the slides were incubated in 3% BSA for 30 min at room temperature to block nonspecific binding. Subsequently, the slides were incubated overnight at 4°C in a 1:300 dilution of an a-SMA antibody generated in rabbit (ab5694, Abcam), washed with PBS (3 washes of 5 min each), and incubated for 1 h in a 1:200 dilution of an anti-rabbit secondary antibody (Servicebio) at room temperature. After washing with PBS 3 times (5 min each), DAB (Liquid DAB + substrate chromogen system, K3468; Dako) was applied for 15 min at room temperature. The slides were washed with running water, counterstained with hematoxylin, washed, dehydrated, and sealed at the edges. Six images per slide (20X magnification) of the muscularis regions were taken under a Nikon Eclipse CI microscope and captured with a Nikon DS-U3 camera.

Smooth muscle cells were identified by specific staining with antibodies against a-SMA. We analyzed the fraction of smooth muscle cells in the nonvascular muscularis in each image using National Institutes of Health Image J software as described by Boreham et al. [21]. Vaginal muscularis (excluding vascular smooth muscle) was outlined manually on each image. The color of *α*-actin–specific staining was identified. The fraction of smooth muscle in the area of interest was determined by computing the area of *α*-actin staining relative to the total area of nonvascular muscularis. Three slides were cut transversely from different portions along the vagina longitudinal axis per animal. Six images were captured per slide. These replicates were averaged per animal and used to obtain the means of each group (n=6 animals/group).

### 2.5. Western Blot Analysis

Protein was extracted from frozen distal vaginal segments (n=6 animals/group) and quantified using a bicinchoninic acid protein assay. The samples were separated by SDS-PAGE (a-SMA, collagen I, and *β*-actin on a 10% gel; collagen III on an 8% gel), and protein was transferred to polyvinylidene difluoride membranes (Millipore, Bedford, Massachusetts). Membranes were blocked with 5% nonfat milk for one hour in 0.5% TBS-T prior to incubation with antibodies. Anti-a-SMA primary antibody (1:2000, ab5694, Abcam), anti-collagen I primary antibody (1:1000, ab34710, Abcam), anti-collagen III primary antibody (1:7000, ab7778, Abcam), anti-*β*-actin primary antibody (1:3000, GB12001, Servicebio), horseradish peroxidase-conjugated goat anti-rabbit IgG secondary antibody (1:3000, GB23303, Servicebio), and horseradish peroxidase-conjugated goat anti-mouse IgG secondary antibody (1:3000, GB23301, Servicebio) were diluted in TBS-T. Immunoreactive bands were visualized by enhanced chemiluminescence (Amersham Pharmacia Biotech). The densitometry of the immunoreactive bands on the Western blot was calculated using Image J software.

### 2.6. Biomechanical Testing

Because we did not expect the biomechanical properties of the vaginal wall to be affected after short-term estrogen withdrawal, we only performed uniaxial biomechanical testing in the control group (Group 1, n=6 animals) and the group after long-term bilateral ovariectomy (Group 4, n=6 animals). Before the testing, the samples were allowed to reach room temperature. To ensure a uniform stress and strain distribution, we cut the samples into a dog-bone shape with an aspect ratio of 5 (length/width) within the mid-substance of the tissue. Then, the 5 mm ends of each sample were gripped using specially designed soft-tissue clamps. The sample-clamp complex was attached to a uniaxial tensile testing machine (Instron™) and preloaded to 1 Newton. Subsequently, the tissue cross-sectional area within the mid-substance of the tissue and the initial clamp-to-clamp distance were measured using a micrometer system. The samples were hydrated throughout the preparation process using 0.9% saline solution. We did not perform cyclic preconditioning prior to the load to failure test. Then, the sample-clamp complex was stretched at a constant deformation rate of 12 mm/min. The load (Newtons) and elongation (millimeters) were recorded. The data points were collected every 0.02 seconds and then imported for analysis to Excel (Excel, Microsoft Corp, Redmond, WA).

A load-elongation curve was generated for each test. The following parameters describing the mechanical properties of the tissue were obtained from this curve: ultimate load at failure (N) and maximal distension (mm). Ultimate load at failure defines the point of tissue disruption on the load-elongation curve and is a measure of the maximum sustainable force of the tissue. Maximal distension is the distension that corresponds to the ultimate load and describes the distance the tissues could be pulled before tissue disruption. A corresponding stress–strain curve was plotted based on the load-elongation curve. The nominal stress (MPa, where 1 Pa=1 N/mm^2^) was calculated by dividing the force (N) by the initial cross-sectional area (mm^2^), and the strain was calculated by dividing the distension (mm) by the initial clamp-to-clamp distance (mm). We analyzed the tangent modulus (MPa) derived from this curve in the linear region. The tangent modulus, which is an indicator of tissue stiffness on a per unit basis, was the maximum slope of the stress–strain curve recorded over a 1% interval of strain.

### 2.7. Statistical Analysis

The data were not normally distributed. To obtain the results of the histological and biochemical analyses, we used a nonparametric analysis, i.e., Kruskal–Wallis ANOVA, and post hoc tests to pairwise compare the groups (Bonferroni correction). In addition, we compared the biomechanical test results of the control group with the 16 weeks' group using a Mann-Whitney U test. A P-value<0.05 was considered statistically significant. All statistical analyses were performed using SPSS version 24.0 (IBM Corp, Armonk, NY).

## 3. Results

### 3.1. Atrophied Vaginal Wall after Ovariectomy

Masson trichrome staining was performed to examine the morphology of the proximal segment in the anterior vaginal wall. Similar to humans, the histological structure of rats comprises the following four layers: epithelium, collagen-rich lamina propria, muscularis containing smooth muscle, and adventitia. Compared with the control group, evident atrophy in the epithelium was observed after ovariectomy, especially at 16 weeks (Figure 1). In addition, the smooth muscle bundles were smaller and poorly organized in the rats with surgically induced menopause.

### 3.2. Collagen Composition and Alignment in the Lamina Propria Differs after Ovariectomy

Sirius Red birefringence was used to assess the collagen alignment in the lamina propria layer of the rat vagina (Figure 2(a)). Under polarizing filters, the collagen fibers showed a mixed proportion of birefringent staining patterns ranging from green and yellow to orange/red, depicting immature (greater likelihood of containing collagen type III) to mature (greater likelihood of containing collagen type I) collagen fibrils, respectively [20]. In the control group, collagen exhibited weak birefringence, appearing thin, greenish, and more scattered. The collagen composition underwent dynamic changes from 2 weeks after ovariectomy, with denser collagen alignment and increasing deposition of thick collagen (orange/red colored). The percent area of mature collagen fibrils in the lamina propria layer was significantly increased after ovariectomy (P<0.001) (Figure 2(b)), while the percent area of immature collagen fibrils was significantly decreased 16 weeks after ovariectomy (P<0.001) (Figure 2(c)).

### 3.3. Smooth Muscle Content in the Proximal Vaginal Wall Muscularis

The morphology and quantity of the nonvascular smooth muscle content in the muscularis of the proximal vaginal wall were identified by specific staining with antibodies against a-SMA as described in the methods section (Figure 3(a)). After ovariectomy, the smooth muscle bundles appeared disorganized, and the fraction of cells positive for a-SMA relative to the entire area of the muscularis was significantly decreased (P<0.001) (Figure 3(b)), especially 16 weeks after ovariectomy (Group 4).

### 3.4. Expression of Collagen Subtypes I/III and a-SMA in the Distal Vaginal Segments

Compared with the control group, collagen I expression was increased after ovariectomy, with a significant increase after 16 weeks (P=0.029) (Figure 4(a)). Although there was a trend towards decreased collagen III expression after ovariectomy, the difference did not achieve statistical significance (P=0.348) (Figure 4(b)). The expression of a-SMA showed no significant differences among any of the groups (P=0.844) (Figure 4(c)).

### 3.5. Biomechanical Properties

The uniaxial biomechanical results of the rats in the normal group and the rats 16 weeks after bilateral ovariectomy are presented in Table 1. All load-elongation curves generated in this study were nonlinear with the characteristic toe, linear, and failure regions. The ultimate load at failure showed a declining trend over 16 weeks after bilateral ovariectomy (9.70±1.42 N in Group 4 versus 12.31±3.50 N in Group 1), but the difference was not statistically significant (P=0.190). There was no significant difference in the maximal distension between the two groups (P=0.905). The tangent modulus was significantly increased after ovariectomy (P=0.016).

## 4. Discussion

POP is a common disease in adult women worldwide. Although menopause is a major risk factor for POP [15, 22], knowledge regarding the effect of menopause on the vaginal wall structure and function and whether such changes can dispose women to develop POP is limited. Therefore, we conducted a comprehensive analysis of rat vaginal wall changes by combining histological, biochemical, and biomechanical analyses both short- and long-term after surgically inducing menopause. In this study, we used an experimental rat model of surgically induced menopause through bilateral ovariectomy to form permanent anestrus [17, 19]. A previous study found that age had a significant effect on the response of the vagina and its supportive tissues to ovariectomy such that ovariectomy significantly affected these tissues in young rats but not in middle-aged rats [23]. Nine-month-old rats are considered middle-aged, approaching ovarian senescence with prolonged cycles [23]. Thus, to clearly clarify the effect of surgically induced menopause on the vaginal wall, we chose young rats (3-6 months) to best reflect the effect of sex hormone withdrawal on the vaginal wall.

The histological analysis in our study revealed that the structural properties of the vaginal wall, including the epithelium, lamina propria, muscularis, and adventitia layers, are similar between rats and humans, thus providing a foundation for observing the impact of menopause on the vaginal wall. Mocan-Hognogi et al. proved that surgically induced anestrus started 15 days after bilateral ovariectomy by detecting significantly decreased estradiol levels after surgery [19]. We also found that the epithelium began to atrophy 2 weeks after ovariectomy, which is consistent with previous studies [24, 25]. In addition, the histological properties of the rat vaginal wall underwent constant changes after ovariectomy, and the most evident atrophy in the epithelium was observed 16 weeks after the surgery in our study. This result may be caused by increased epithelial cell apoptosis resulting from estrogen withdrawal [24].

Vaginal smooth muscle is essential for the maintenance of the vaginal tone and overall compliance of the vagina. Smooth muscle attaches the vagina to the levator ani muscles and plays an important role in pelvic organ support [26]. Previous studies have demonstrated that the fraction of smooth muscle in the muscularis in prolapsed vaginal tissues was decreased, which may be involved in the pathophysiology of POP [11, 21]. Our results showed that the smooth muscle bundles in the proximal vaginal wall were disorganized and that the fraction of smooth muscle in the muscularis was significantly decreased from 2 weeks after ovariectomy. Berman et al. reported similar results [24]. In contrast, estradiol treatment induced significant increases in smooth muscle in the vaginal muscularis [27]. However, we did not find a decrease in the fractional area of smooth muscle within the muscularis in the distal vaginal after ovariectomy. The different findings between the proximal and distal vagina may be due to the different methods applied to detect the smooth muscle content. Furthermore, the proximal vagina is differentiated from the mesoderm, while the distal vagina is differentiated from the ectoderm [28]. Regional differences in the vaginal muscularis have been reported between the proximal and distal vagina [29]. Thus, the different reactions to estradiol withdrawal may be due to the different embryological origins of the proximal and distal vagina, which deserves further research.

Fibrillar collagen I and collagen III are the predominant components of the extracellular matrix and play essential roles in the maintenance of vaginal support [30]. In this study, we quantified the collagen subtypes using both histological and biochemical methods and obtained consistent results. In normal rats, the predominant collagen subtype in the anterior vaginal wall is collagen III, which is consistent with the results reported by Moalli et al. [12]. Collagen in the vagina undergoes continuous remodeling throughout life, including during pregnancy, during parturition, and after menopause. Estrogen withdrawal not only induces marked changes in the vaginal collagen subtypes but may also play an important role in the pathogenesis and progression of POP [27]. We found that collagen I was significantly increased from 2 weeks after ovariectomy, while collagen III showed a declining trend. The metabolism and response to menopause status of the extracellular matrix of the rat vagina may differ from those in humans. In our study, the fraction of smooth muscle in the muscularis of the proximal vaginal wall was significantly decreased from 2 weeks after ovariectomy, which could decrease the biomechanical strength. We hypothesize that the increased synthesis of collagen I, which provides tensile strength and stiffness, may be a compensatory mechanism that counteracts the decrease in smooth muscle. We aim to further study the molecular mechanisms of the effect of ovarian hormones on the structure components of the rat vagina.

In this study, we conducted a uniaxial loading test to characterize the biomechanical properties of the anterior rat vagina. We found that surgically induced menopause led to long-term changes in the structural components (including collagen subtypes and smooth muscle) and, subsequently, the mechanical properties of the rat vagina. Mechanically, the vagina requires a minimum stiffness and strength to meet the demands of physiological loading. The lamina propria and muscularis layers contribute to both the viscoelasticity and strength of the vagina. The different diameters of collagen I and collagen III may account for the different mechanical properties with thinner collagen fibers contributing to lower stiffness [31]. In addition, a reduction in the smooth muscle content in the vaginal muscularis may impair vaginal tone and contractility [11]. In our study, the higher stiffness levels (tangent modulus) may be due to the increased expression of collagen I and denser collagen alignment in the lamina propria, while the reduced smooth muscle content in the proximal vagina may account for the declining trend in the ultimate load at failure in the vagina of the surgically induced menopause rats. Moalli et al. [23] found that ovariectomy could induce a 40% decrease in linear stiffness in pelvic tissues in young and aged rats. However, these authors tested the vagina and its supportive tissues (including the paravaginal attachments to the pelvic sidewall, uterosacral ligaments, and perineal membrane) as a complex in biomechanical testing. In addition, these authors did not further study the changes in the structural proteins in the rat vagina and its supportive tissues, such as collagen and elastin, after ovariectomy. Thus, comparing the study conducted by Moalli et al. and our study is difficult. Similar to our results, Montoya et al. found that low-dose vaginal estrogen treatment resulted in a robust disproportionate increase in collagen type III mRNA in a menopausal rat model, which contributed to the decrease in vaginal stiffness [18]. However, we preloaded all of the samples to 1 N in this study, which was large for the samples with a lower ultimate load at failure. This preloading may affect the load to failure test of these samples because of the potential for plastic deformation.

Several studies have evaluated vaginal tissue from women with and without POP and found that prolapsed vaginal walls express significantly less collagen III and have higher stiffness than control tissue [9, 32, 33]. In this study, we demonstrated that surgically induced menopause had significant short- and long-term impact on tissue composition of the rat vagina, which may impair the biomechanical properties and thereby lead to increased susceptibility to POP development. Further investigation is needed to specifically examine if parallel changes happen in the vaginal wall of postmenopausal women.

## 5. Conclusion

In this study, we showed that the rat anterior vaginal wall underwent continuous changes in collagen subtypes and smooth muscle content from 2 weeks after ovariectomy, including increased expression of collagen I, decreased expression of collagen III, and reduced fraction of smooth muscle in the proximal muscularis. Compared with the control group, the anterior vaginal wall exhibited a higher tangent modulus and a decreasing trend in the ultimate load at failure 16 weeks after ovariectomy. The ovariectomized rat model improved our understanding of the contribution of menopause to the pathogenesis of prolapse.

## Figures and Tables

**Figure 1:** Representative images (×100) of Masson trichrome staining of the (E) epithelium, (LP) lamina propria, (M) muscularis, and (Ad) adventitia at the proximal segment of the anterior vaginal wall. (a) Group 1: control group; (b) Group 2: 2 weeks after ovariectomy; (c) Group 3: 4 weeks after ovariectomy; (d) Group 4: 16 weeks after ovariectomy. (a) shows normal histological structures; (b), (c), and (d) show evident epithelium atrophy and smaller and poorly organized smooth muscle bundles. Scale bar=100 *μ*m.

**Figure 2:** Collagen composition and alignment of the lamina propria layer in the rat vaginal wall. (a) Birefringence images (×200) of Sirius Red-stained tissues showing Group 1 (control group), Group 2 (2 weeks after ovariectomy), Group 3 (4 weeks after ovariectomy), and Group 4 (16 weeks after ovariectomy). The percent area of mature collagen (b) and immature collagen (c) within the lamina propria in the four groups. The data are presented as the mean±SEM of n=6 animals/group. Scale bar represents 100 *μ*m. Significant differences (P<0.05) are denoted (*∗*).

**Figure 3:** Morphology and quantity of the nonvascular smooth muscle content in the muscularis of the proximal vaginal wall. (a) Immunohistochemistry images (×200) of a-SMA: Group 1 (control group), Group 2 (2 weeks after ovariectomy), Group 3 (4 weeks after ovariectomy), and Group 4 (16 weeks after ovariectomy). The fractional area of smooth muscle in the muscularis in the four groups (b). The data are presented as the mean±SEM of n=6 animals/group. Scale bar represents 100 *μ*m. Significant differences (P<0.05) are denoted (*∗*). Ep: epithelium, M: muscularis.

**Figure 4:** Protein expression of collagen subtypes I/III and a-SMA in the distal segments of the anterior vaginal wall. Representative Western blots of (a) Collagen I, (b) collagen III, and (c) a-SMA. Protein expression was normalized to *β*-actin. G1: Group 1 (the control group), G2: Group 2 (2 weeks after ovariectomy), G3: Group 3 (4 weeks after ovariectomy), G4: Group 4 (16 weeks after ovariectomy). The data are presented as the mean±SEM of n=6 animals/group. Significant differences (P<0.05) are denoted (*∗*).

**Table 1:** Comparison of the biomechanical properties of ultimate load at failure, maximal distension and tangent modulus in the linear region between group 1 (control group) and group 4 (16 weeks after ovariectomy).

	Group 1 (n=6)	Group 4 (n=6)	P-value
Ultimate load at failure (N)	12.31±3.50	9.70±1.42	0.190
Maximal distension (mm)	67.68±20.11	61.98±17.47	0.905
Tangent modulus (MPa)	0.25±0.11	0.74±0.27	0.016

^a^Mann-Whitney U test. The data are presented as the mean±standard deviation.

## Data Availability

The data used to support the findings of this study are included within the article.
